The article "Up-Regulation of Intestinal Epithelial Cell Derived IL-7 Expression by Keratinocyte Growth Factor through STAT1/IRF-1, IRF-2 Pathway" was retracted in 2024. Reasons: errors in the text; original data or images not available; unreliable results or conclusions; concerns about the images.

# Up-Regulation of Intestinal Epithelial Cell Derived IL-7 Expression by Keratinocyte Growth Factor through STAT1/IRF-1, IRF-2 Pathway

**DOI:** 10.1371/journal.pone.0058647

**Published:** 2013-03-12

**Authors:** Yu-Jiao Cai, Wen-Sheng Wang, Yang Yang, Li-Hua Sun, Daniel H. Teitelbaum, Hua Yang

**Affiliations:** 1 Department of General Surgery, Xinqiao Hospital, Third Military Medical University, Chongqing, China; 2 Department of Surgery, The University of Michigan Medical School, Ann Arbor, Michigan, United States of America; National Cancer Institute, United States of America

## Abstract

**Background:**

Epithelial cells(EC)-derived interleukin-7 (IL-7) plays a crucial role in control of development and homeostasis of neighboring intraepithelial lymphocytes (IEL), and keratinocyte growth factor (KGF) exerts protective effects on intestinal epithelial cells and up-regulates EC-derived IL-7 expression through KGFR pathway. This study was to further investigate the molecular mechanism involved in the regulation of IL-7 expression by KGF in the intestine.

**Methods:**

Intestinal epithelial cells (LoVo cells) and adult C57BL/6J mice were treated with KGF. Epithelial cell proliferation was studied by flow cytometry for BrdU-incorporation and by immunohistochemistry for PCNA staining. Western blot was used to detect the changes of expression of P-Tyr-STAT1, STAT1, and IL-7 by inhibiting STAT1. Alterations of nuclear extracts and total proteins of IRF-1, IRF-2 and IL-7 following IRF-1 and IRF-2 RNA interference with KGF treatment were also measured with western blot. Moreover, IL-7 mRNA expressions were also detected by Real-time PCR and IL-7 protein level in culture supernatants was measured by enzyme linked immunosorbent assay(ELISA).

**Results:**

KGF administration significantly increased LoVo cell proliferation and also increased intestinal wet weight, villus height, crypt depth and crypt cell proliferation in mice. KGF treatment led to increased levels of P-Tyr-STAT1, RAPA and AG490 both blocked P-Tyr-STAT1 and IL-7 expression in LoVo cells. IRF-1 and IRF-2 expression *in vivo* and *in vitro* were also up-regulated by KGF, and IL-7 expression was decreased after IRF-1 and IRF-2 expression was silenced by interfering RNA, respectively.

**Conclusion:**

KGF could up-regulate IL-7 expression through the STAT1/IRF-1, IRF-2 signaling pathway, which is a new insight in potential effects of KGF on the intestinal mucosal immune system.

## Introduction

Intestinal epithelial cells (IECs) function as active participants in local immune regulation via secreting a variety of cytokines. Among these, interleukin-7 (IL-7) is particularly important in terms of its pleiotropic function in the intestinal immune system [1]. In the intestine, IL-7 is produced by IECs, and in turn IL-7 receptors (IL-7R) have been detected on intraepithelial lymphocytes (IELs) [2]. Studies have demonstrated that IEC-derived IL-7 stimulates the proliferation of lamina propria lymphocytes and IELs [3], [4] and also enhances cytokine release from these lymphocytes in humans [5]. In addition, IL-7 is essential for early developmental processes such as the differentiation of pre-T cells into mature thymocytes. This latter function cannot be performed by any other known cytokines [6]. In the absence of IL-7, homeostatic proliferation of naive T-cells is almost completely abolished, and the lifespan of naive T cells is greatly reduced [7]. In vivo, our group found administration of IL-7 has been demonstrated to enhance IEL functional capacity and population [8]. Geiselhart et al. [9] reported that IL-7 administration altered the peripheral T cell CD4-to-CD8 ratio and resulted in an increase in peripheral T cell numbers and altered function. Watanabe et al. [4] observed that exogenous IL-7 administered to mice resulted in a stimulation of lamina propria lymphocytes. All these data suggest that IL-7 may be essential for ongoing maintenance of IEL function and growth.

Keratinocyte growth factor (KGF) is produced exclusively by mesenchymal cells and IELs, and acts on epithelial cells [10], [11], through its receptors FGFR, indicating that the intestine can both synthesize and respond to KGF [10], [12], [13]. KGF has been reported to play a critical role in intestinal epithelial growth and maintenance. An interest finding shows, after bone marrow transplantation (BMT), KGF could lead to increased IL-7 production [14], and the protective effects of pre-BMT were improved by KGF administration on thymopoiesis [14]. Our previous study reported KGF could up-regulate IL-7 expression through the KGF-KGFR pathway both in an intestinal ischaemia/reperfusion (I/R) mouse model and in LoVo cells [15]. However, the mechanism by which pathway involved in this regulation of IL-7 expression is still unclear.

STATs are a family of latent cytoplasmic proteins that are involved in transmitting extracellular signals to the nucleus. KGF-stimulated increase in GM-CSF levels in lung tissue, which was associated with STAT5 phosphorylation in alveolar macrophages, was consistent with epithelium-driven paracrine activation of macrophage signaling through the KGF receptor/GM-CSF/GM-CSF receptor/ JAK-STAT axis [16]. Epidermal growth factor (EGF) is another important growth factor contributing to normal homeostasis and healing of the ocular surface [17], [18]. EGF has been reported to mediate its effect on target cells through the JAK-STAT pathway [19]-[20]. We sought to determine whether KGF, similar to EGF, activates this pathway in mediating effects on intestinal epithelial cells.

Interferon regulatory factors (IRFs) are a large family of transcription factors, in which IRF-1 and IRF-2 were first identified as activator and repressor, respectively [21]. The regulation of CIITA pIV by IFN-γ in B cells depends on the binding of signal transducer and activator of transcription (STAT)1 to IFN regulatory factor (IRF)-1 and IRF-2 to an interferon regulatory factor element (IRF-E) [22]. It has also been found that the STAT1 activation of IRF-1 plays an important role of STAT1 in promoter IV activation [23], [24]. Another study showed the transcriptional regulation via an IRF-E was important for IL-7 production in human IECs [1], which is consistent with the previous report on murine keratinocytes[25]. Of note, it was found that not only IRF-1 but also IRF-2, could up-regulate IL-7 production [1].

In this study, we demonstrated for the first time that the KGF signaling pathway was involved in the regulation of IL-7 expression in LoVo cells, and hypothesized that up-regulation of intestinal epithelial cell derived IL-7 expression by KGF through STAT1, IRF-1/IRF-2 pathway. This study would gain a better understanding of the functions of this cytokine on local immune regulation.

## Materials and Methods

### Ethics Statement

The study has been approved by the ethics committee of Xinqiao Hospital, Third Military Medical University. Animals were handled according to the guideline for the care and use of laboratory animals.

### Cell culture

Human intestinal epithelial LoVo Cells (ATCC CCL-229) were used in our experiments. Cells were cultured in Dulbecco's modified Eagle's medium (DMEM) containing 10% fetal calf serum, 50 units/ml penicillin, and 50 mg/ml streptomycin, refreshed every 48 h, and subcultured serially when 80% confluent. Cells were seeded at identical cell densities and were typically used 12–15 days after reaching confluence.

### Cell treatment

Cells were grown on 6-well plates and incubated with Recombinant human KGF (rHuKGF) (150 ng/ml) for 0, 30 min, 1, 2, 3, 6, 48 h, respectively. Then cells were fixed for staining experiments and nuclear extracts or total protein extraction of cells was used for Western blotting detection.

For STAT signaling pathway analysis, inhibitors including rapamycin (RPM) and AG490 were used. The cells were randomly allocated into three groups. Two of the groups were treated with either RPM (50 ng/ml, catalogue no. 37094; Sigma), or AG490 (50 µmol/l, catalogue no. S1509; Sigma) and one group of cells was left untreated as a control. The samples were harvested 24 h after the onset of stimulation for further study.

IRF1 and IRF2 expression were silenced by using interfering RNA and the plasmids 663, 664 and 665 (Shanghai SunBio Medical Biotechnology Co., Ltd) were transfected into LoVo cells for silencing IRF1 and plasmids 691, 692 and 693 (Shanghai SunBio Medical Biotechnology Co., Ltd) for IRF2, respectively, with lipofectamine 2000 (Invitrogen) following the manufacturer's instructions as previously.

### Flow cytometric analysis

LoVe cells were cultured as described above. The amount of BrdU incorporated into the cells was measured following the procedures according to the manual in the kit (Flow Cytometry BrdU Testing Kit, GENMED). Briefly, 1×10^6^ cells were pulse-labeled for 30 min with 10 mM BrdU, washed in ice-cold PBS, and pelleted. Cell pellets were resuspended in PBS and cells fixed in ice-cold ethanol. Incorporation of BrdU was measured with a fluorescein isothiocyanate (FITC, green)-conjugated anti-BrdU antibody and propidium iodide (PI, red). Flow-cytometric analysis was done with BD VERSE (Becton Dickinson) and accompanying BD FACSuite software, with forward and side scatter gates set to exclude nonviable cells.

### Enzyme linked immunosorbent assay(ELISA)

ELISA analysis was used to evaluate the expression of secreted IL-7. For quantification of IL-7 in the supernatant of cultured LoVo cells, conditioned culture media were collected and centrifuged at 1200 rpm for 5 min to remove particulates; cleared supernatant was collected, concentrated, and stored at −80 °C until use. A human IL-7 ELISA Quantikine™ HS (High Sensitivity) from R&D Systems was used for detection of IL-7. The protocol was performed according to the manufacturer's instruction. The absorbance for IL-7 was assayed and the concentrations of each were determined by interpolation against a standard curve.

### Animals

Male, 6-8week-old, specific pathogen-free, C57Bl/6 mice were purchased from Laboratory Animal Center, Third Military Medical University, Chongqing, P.R. China, maintained in temperature, humidity, and light-controlled conditions. Mice were divided into two groups: KGF group and control. Recombinant human KGF (rHuKGF) administration to mice was given daily by intraperitoneal injection (5 mg/kg/ day) for five days. In all experiments, six animals were analyzed per group and three times of experiments were repeated. There was no significant difference in survival between treatment and control groups.

### Histological score

Segments of jejunum were harvested, were fixed with 4% paraformaldehyde and used for histological analysis. Tissues were then dehydrated with ethanol and embedded in paraffin. Sections were cut and stained with hematoxylin-eosin(H&E). Histological changes were assessed by a pathologist in a blinded fashion. Especially, the villus height and depth of crypt were measured using a calibrated micrometer. Each measurement of villus height and crypt depth consisted of the mean of 7 different fields.

### Epithelial Cells Proliferation Assay

Crypt cell proliferation rate was calculated by the ratio of the number of crypt cells incorporating PCNA to the total number of crypt cells. Samples fixed by 4% paraformaldehyde were cut into 8 m-thick sections, treated with 0.5% hydrogen peroxide in methanol solution, blocked for 45 min, and then incubated with an anti-PCNA(catalogue no. 10205-2-AP; Proteinteck) or purified rabbit IgG (10 mg/ml; negative control) overnight at 4°C. The sections were incubated with biotinylated goat antirabbit IgG for 60 min and reacted with streptavidin-enzyme conjugates (Vector Laboratories Inc), and then the peroxidase activities were developed by diaminobenzidin. The total number of proliferating cells per crypt was defined as a mean of proliferating cells in 10 crypts (Original magnification ×400).

### Mucosal wet weight, RNA and protein measurements

At the time of death, 10 cm of jejunum was excised and this segmental of intestine was weighed and was used for the measurement of intestinal RNA and protein content. Intestinal mucosal RNA was determined by spectrophotometry using a modified Schmidt-Tannhauser method as described by Munro and Fleck [26]. Protein determination was performed by using a Bio-Rad protein assay kit (Bio-Rad Laboratories, Hercules, CA). RNA is expressed in µg/cm segment of intestine and protein results are expressed in mg/cm segment of intestine.

### RNA Isolation, Reverse Transcriptase, and Polymerase Chain Reaction(PCR)

Total RNA specimens were isolated by using the Trizol reagents (catalogue no. 15596026; Invitrogen). Total RNA was reverse transcribed into cDNA using SuperScript II H-reverse transcriptase (catalogue no. 18064071; Invitrogen). PCR amplification primers of IL-7 were as follows: Up 5-TCTAATggTCAgCATCgATCA-3 and Down 5-gTggAgATCAAAATCACCAgT-3; Taqman probe was 6FAM-CCgCCgCCCgTCCACACCCgCCph, as described previously [27]. Amplification standard curves of target genes and of the reference gene β-actin were established, as previously described [27]. A PCR reaction mixture (30 µL) containing 1 mM dNTP (Life Technologies), 0.3 µM of each oligonucleotide primer, 1 µM Taqman probe, 1 U AmpliTaqGold DNA polymerase (Roche, Branchburg, NJ), and 100 ng of sample cDNA in PCR buffer was amplified on an ABI Prism 7700 sequence detector (Applied BioSystems). Cycling conditions included initial denaturation at 94 °C for 10 minutes, 30 seconds at 94 °C, 30 seconds at 60 °C, and 45 seconds at 72 °C for 45 cycles. All assays were performed in triplicate. The quantities of IL-7 gene expression and of the reference gene β-actin were determined by using standard curves. The mRNA copy numbers of these targets were calculated for each sample from the standard curve by measuring the threshold cycle value. The target amount was then divided by the reference gene amount to obtain a normalized target value and presented as relative rates compared with the expression of the reference gene β-actin.

### Western blot assay

The nuclear extracts and total proteins were prepared from treated LoVo cells, as described previously [28]. Protein concentrations were measured, and equal amounts of nuclear extracts or total proteins were fractionated on 10% SDS polyacrylamide gel and transferred to 0.2-µm nitrocellulose membrane. Nitrocellulose blots were blocked by incubation in TBST (10 mM Tris-HCl, pH 7.5, 150 mM NaCl, and 0.1% Tween 20) containing 5% milk for 1 h. Blots were incubated with appropriate antibodies against IL-7(catalogue no. ab-9628; Abcam Inc.), IRF-1 (catalogue no. sc-13041; Santa Cruz Biotechnology), IRF-2 (catalogue no. sc-13042; Santa Cruz Biotechnology), STAT1 (catalogue no. 10144-2-AP; Proteinteck), or P-Tyr-STAT1 (Tyr701) (catalogue no. 7649; Cell Signaling Technology). After washed, the membrane was incubated with HRP-conjugated secondary antibodies (Cell Signaling) and then visualized with enhanced chemiluminescence (Cell Signaling). β-tubulin (Sigma, Dorset, UK) was used as an internal control.

### Immunofluorescence staining

Cells and sections were fixed for staining experiments. Cells were incubated with the following primary antibodies: anti-IRF-1 rabbit polyclonal antibody (catalogue no. sc-13041; Santa Cruz Biotechnology) and anti-IRF-2 rabbit polyclonal antibodies (catalogue no. sc-13042; Santa Cruz Biotechnology) and sections were incubated with anti-IL-7 rabbit polyclonal antibody (catalogue no. bs-1811R; Beijing Boisynthesis Biotechnology Co.,Ltd.) overnight at 4C. Then the cells and sections were stained with FITC-conjugated goat anti-rabbit IgG. Nuclear staining for total cell counting was performed by 5 min addition of 1 mg/ml of DAPI (40,60-diamidino-2-phenylindole) and the fluorescence signals were analyzed by recording and merging single-stained images, using confocal laser microscope (Leica TCS SP2). Images were processed using Adobe Photoshop (Adobe Systems, San Jose, Calif., USA) and was analyzed by Leica's software system.

### Immunohistochemistry staining

Samples fixed by 4% paraformaldehyde were incubated with either an anti-IRF-1 (catalogue no. sc-13041; Santa Cruz Biotechnology) antibody, an anti-IRF-2 (catalogue no. sc-13042; Santa Cruz Biotechnology) antibody or purified rabbit IgG (10 mg/ml; negative control). After the samples were counterstained with hematoxylin, the localization of IRF-1, IRF-2 was examined by light microscopy (Original magnification ×400).

### Statistical analysis

Data are expressed as means ± standard deviation (SD). Statistics were performed using SPSS 13.0 software. Results were analyzed using analysis of variance (ANOVA). Statistical significance was defined as *P*<0.05.

## Results

### KGF administration leads to EC proliferation both *in vivo* and *in vitro*

#### Proliferation in a cell culture model

To investigate if the LoVo cells were proliferated after KGF treatment, we analyzed BrdU-incorporation expression by using flow cytometry. Results showed LoVo cells treated with KGF at different concentrations (0, 80 and 150 ng/ml) for 48 h displayed BrdU+ population increased to 26.9% and 31.1% with treatment of KGF (80 and 150 ng/ml, respectively) compared with control (12.0%), suggesting that cell viability was induced by KGF (Figure 1).

**Figure 1:** Detection of cell viability by flow cytometric analysis of BrdU-incorporation. Incorporation of BrdU was measured with a fluorescein isothiocyanate (FITC, green)-conjugated anti-BrdU antibody and propidium iodid (PI, red), shows a typical example of flow cytometric analysis of LoVo cells proliferation after KGF treatment, where a BrdU+ population is clearly visible. Control (A), KGF treated groups with different concentrations including 80 ng/ml (B) and 150 ng/ml (C).

#### Intestinal Morphology

To investigate the effect of KGF on mice intestinal mucosa, histopathological evaluation was used. There was a significant increase in both villus height and crypt depth in the group after KGF treatment. KGF treatment led to an increase in jejunal villus height 387±49 µm), as compared with control (243±42 µm) (P<0.05). The crypt depth was also greater in the KGF group (116±21 µm) than in control (53±17 µm) (P<0.05), respectively (Figure 2).

**Figure 2:** Alterations in villus height and crypt depth in mice after KGF treatment. * *P*<0.05 vs. control group, n = 6 per group.

PCNA-positive cells were all distributed in the crypt of Lieberkuhn of the small intestine. KGF also significantly increased the number of PCNA positive cells to (57.2±5.4%) when compared with control (23.7±3.9%) (P<0.05) (Figure 3). There was no significant difference in the positions of positive cells between groups, and all positive cells remained in the crypts.

**Figure 3:** Alterations in PCNA expression in small intestine of KGF treated mice by immunohistochemistry. PCNA expression was significantly increased in KGF group (A), as compared to the control group (B). PCNA expression is expressed as means ± SD (C), *P<0.05 vs control group. Original magnification: ×400; n = 6 per group. Scale bar = 25 µm

#### Indexes of jejunum

Mucosal wet weight of the jejunum (mg/10 cm) was significantly increased in KGF group compared with the control. KGF administration significantly increased RNA content (39.7±6.4 µg/cm) when compared with control (16.2±4.5 µg/cm) (P<0.05). The changes of jejunum mucosal protein contents were similar to changes of RNA content. There was significant difference of protein contents between the KGF group (2.65±0.19 mg/cm) and the control group (1.78±0.26 mg/cm) (P<0.05) (Table 1).

**Table 1:** Intestinal wet weight and contents of jejunal protein and RNA.

	Control	KGF group
Protein (mg/cm)	1.78±0.26	2.65±0.19*
RNA (µg/cm)	16.2±4.5	39.7±6.4*
Intestinal wet weight (mg/10 cm)	387.8±8.4	576.4±11.7*

* *P*<0.05 vs Control group.

### KGF administration results in an increased expression of EC -derived IL-7 both *in vivo* and *in vitro*

To investigate the role of KGF in the regulation of IL-7, both *in vitro* and *in vivo* models were used. KGF administration at different concentrations (20, 40, 80, 100 and 150 ng/ml) for 48 h in the LoVo cells resulted in an increased IL-7 expression detected by Western blot assay, showing a dose-dependent manner [15], which was also confirmed by ELISA. We found that IL-7 levels in cell culture supernatant rose from 4.43±0.47, 5.52±0.41, 6.47±0.45, 8.72±0.53 pg/mL in the KGF (20, 40, 80,150 ng/ml) treated group to 2.33±0.28 pg/mL in the control. Furthermore, IL-7 expression in the intestinal mucosa was dramatically increased in protein nearly 4-folds compared with control in a health mouse model [15]. Moreover, KGF up-regulated IL-7 in a mouse model of intestinal I/R, which was confirmed by the results from immunofluorescence staining [15].

### STAT1 pathway is involved in the regulation of IL-7 after KGF treatment

#### KGF treatment leads to increased levels of P-Tyr-STAT1

To gain direct evidence for the activity of the STAT1 signaling pathway induced by KGF in LoVo cells, the STAT1 activity was evaluated by Western blot analysis (Figure 4). Compared with control cells, KGF (150 ng/ml) treatments of different time point (30 min, 1, 2, 6 and 24 h) resulted in significantly increased levels of P-Tyr-STAT1 (P<0.05) (Figure 4), but not STAT1 proteins at all time points including 30 min, 1 h, 2 h, 6 h and 24 h.

**Figure 4:** Changes of P-Tyr-STAT1 and STAT1 expression after KGF treatment in LoVo cells. Increased expression of P-Tyr-STAT1, but not STAT1, were confirmed by western blot in LoVo cells with KGF (150 ng/ml) treatment. Tubulin was used as internal control.

#### To inhibit STAT1 expression causes a significant down-regulation of IL-7 expression in LoVo cells

Both RAPA and AG490 are inhibitors of STAT1. The effects of RPM or AG490 on STAT1 and IL-7 protein expression were determined by Western blot analysis (Figure 5A). The results showed that the protein levels of P-Tyr-STAT1 and IL-7 were significantly decreased by the treatment with RPM or AG490 partially counteracted the effects of KGF, while STAT1 proteins did have not significantly decreased when compared with the control (P<0.05) (Figure 5A). Similarly, we analyzed the IL-7 mRNA expression by using quantitative real-time PCR. The results were shown in Figure 5B, which were similarly to IL-7 protein expression.

**Figure 5:** Changes of P-Tyr-STAT1, STAT1 and IL-7 expression after STAT1 blockade following KGF treatment, by western blot in LoVo cells (A). Tubulin was used as internal control. Suppressions of P-Tyr-STAT1 and IL-7 expression, but not STAT1, were observed with STAT1 inhibitors including AG490 (50 µmol/l) and RPM (50 ng/ml) following KGF (150 ng/ml) treatment. Changes of IL-7 mRNA expression after STAT1 blockade following KGF treatment were detected by quantitative real-time PCR (B), * indicates significant difference between RPM (or AG490) group and control, ** indicates significant difference between RPM (or AG490)+KGF group and control+KGF group, P<0.05.

### IRF-1 and IRF-2 are involved in the up-regulation of IL-7

This study showed the evidence for the activity of the STAT1 signaling pathway induced by KGF, and the previous report found that the transcriptional regulation via an IRF-E including IRF-1 and IRF-2, was important for IL-7 production in human IECs [1], which suggest IRF-1 and IRF-2 are involved in the regulation of IL-7.

#### KGF treatment results in an increased expression of IRF-1 and IRF-2 both in vivo and in vitro

To further investigate the pathway involved in this regulation of IL-7 expression, LoVo cells were treated with KGF (150 ng/ml) for 0 h, 2 h, 3 h and 6 h, and IRF-1, IRF-2 expressions of the nuclear extracts and total proteins were detected by Western blot. Results showed a significantly increased IRF-1 and IRF-2 expression in 6 h both in nuclear extracts and total proteins respectively; *P*<0.05 compared with controls) (Figure 6A, 6B). These results were confirmed with another finding, which showed that LoVo cells were treated with KGF (150 ng/ml), for 0 h, 1 h, 3 h and 6 h, and immunofluorence staining was performed to detect the expressions of IRF-1, IRF-2 in the nucleus. Results showed the fluorescence band of IRF-1 and IRF-2 in nuclear, which were most obvious at 6 h than other time points in LoVo cells (Figure 7A, 7B). All these results suggest that KGF treatment caused increased expressions of IRF-1 and IRF-2 with a time dependent manner (Figure 6A, B, 7A, B).

**Figure 6:** KGF administration resulted in an increased IRF-1 and IRF-2 expression of the nuclear extracts and total proteins in vitro. Dose-dependent increased expression both of IRF-1 (A) and IRF-2 (B) were confirmed by western blot in LoVo cells with KGF treatment. Tubulin and H1 were used as internal control.

**Figure 7:** Increased expression of IRF-1 and IRF-2 were confirmed by immunofluorenscence staining with KGF treatment in vitro. Increased expression of IRF-1 and IRF-2 in the nucleus were observed after 6 h with KGF treatment.

Immunohistochemistry was done to detect the IRF-1 and IRF-2 expression 5 days after KGF administration in a mouse model. Results showed that KGF administration also increased the number of positive cells which express IRF-1 and IRF-2 preferentially exhibited nuclear patterns, indicating that these IRF proteins function as transcriptional regulators in IECs in vivo (Figure 8). Furthermore, the number of the IRF-2-positive cells was much more than IRF-1 -positive cells (Figure 8). These findings were consistent with our present report *in vitro*. Recombinant KGF acts on the intestinal epithelial cells leading to the up-regulation of IRF-1 and IRF-2 expressions and subsequent IL-7 expression.

**Figure 8:** Alterations in IRF-1 and IRF-2 expression in small intestine of KGF treated mice by immunohistochemistry. IRF-1 expression in control group (A) and in KGF group (B), IRF-2 expression in control group (C) and in KGF group (D). Original magnification: ×400; n = 6 per group. Scale bar = 25 µm.

#### Changes of IL-7 expression after IRF-1 and IRF-2 expression were silenced

To further confirm the pathway of KGF through IRF-1 and IRF-2 to regulate IL-7 expression, IRF-1 and IRF-2 expression were silenced by using interfering RNA, and then the effect of KGF on the IL-7 expression was investigated in the LoVo cells. The IL-7 protein and mRNA expression was determined by Western blot analysis and quantitative real-time PCR. The plasmids 663, 664 and 665 used for IRF-1, plasmids 691, 692, 693 for IRF-2 were transfected into LoVo cells and the IRF-1 and IRF-2 expression of the nuclear extracts and total proteins were detected by Weston blot, respectively. Results showed the IRF-1 expression, both in the nuclear extracts and total proteins, were dramatically reduced, when treated with 665 plasmid, compared to controls (p<0.05), while the same condition was found in IRF-2 expression (treated with 693 plasmid) compared to controls, p<0.05) (Figure 9A, 9B). Following IRF-1 silencing by plasmids 665 and IRF-2 silencing by plasmids 693, LoVo cells were treated with 150 ng/ml KGF for 48 h, respectively and significant reduction of IL-7 expression were noted. IL-7 protein expression significantly reduced by treated with 665 plasmid for IRF-1(p<0.05) and by treated with 693 plasmid for IRF-2 (p<0.05), compared to control, respectively (Figure 9C, 9D), which were also found in IL-7 mRNA expression detected by quantitative real-time PCR. These results showed that transfection of plasmid 665 and plasmid 693 could result in obvious suppression of IRF-1 and IRF-2 expression respectively, so that decreased IL-7 expression was observed in LoVo cells following KGF treatment. However, transfection of control plasmid had no influence on the mRNA and protein expression of IL-7. These findings further confirm that KGF can regulate IRF-1 and IRF-2 expressions and subsequent IL-7 expression in IECs.

**Figure 9:** IL-7 is up-regulated by KGF through IRF-1/IRF-2 pathway. Tubulin and H1 were used as internal control. (A) Reduced the nuclear extracts and total proteins of IRF-1 was confirmed by western blot in LoVo cells following IRF-1 RNA interference. Plasmids 663, 664 and 665 were transfected into LoVo cells and IRF-1 expression was detected. Plasmid 665 can definitely inhibit IRF-1 expression. (B) Reduced the nuclear extracts and total proteins of IRF-2 was confirmed by western blot in LoVo cells following IRF-2 RNA interference. Plasmids 691, 692 and 693 were transfected into LoVo cells and IRF-2 expression was detected. Plasmid 693 can definitely inhibit IRF-2 expression. (C) Reduced expression of IL-7 was confirmed by western blot and quantitative real-time PCR in LoVo cells following IRF-1 RNA interference. Decreased expression of IL-7 was observed in LoVo cells following KGF treatment in response to RNA interference of IRF-1 by plasmid 665 in both mRNA and protein levels. *P<0.05 vs. control group. (D) Reduced expression of IL-7 was confirmed by western blot and quantitative real-time PCR in LoVo cells following IRF-2 RNA interference. Decreased expression of IL-7 was observed in LoVo cells following KGF treatment in response to RNA interference of IRF-2 by plasmid 693 in both mRNA and protein levels. *P<0.05 vs. control group.

## Discussion

In this study, we found that KGF administration resulted in EC proliferation both *in vivo* and *in vitro* study. KGF treatment led to increased levels of P-Tyr-STAT1, and RAPA and AG490 both blocked P-Tyr-STAT1 and IL-7 expression in LoVo cells. KGF also up-regulated IRF-1 and IRF-2 *in vivo* and *in vitro* studies, and IL-7 expression was decreased after IRF-1 and IRF-2 expression was silenced by using interfering RNA in LoVo cells, respectively. All these results suggest that KGF could up-regulate the IL-7 expression through the STAT1/ IRF-1, IRF-2 signaling pathway.

It is believed that KGF plays a critical role in intestinal epithelial growth and maintenance [29]. Our present study showed that KGF administration led to proliferation in LoVo cells, and also found that there was a significant increase in villus height, crypt depth and the number of PCNA positive cells in mice after KGF treatment. In addition, KGF significantly increased the intestinal mucosal wet weight, RNA and protein contents. These results suggested the important role of KGF in the intestinal epithelial growth, which was confirmed by the study of Farrell *et al* [30], who found that wet weights of the intestinal segments were increased by the KGF treatment and morphometric measurement showed that both crypt depth and villus height were also increased in mice.

Recent studies have demonstrated that the interactions between intestinal EC and mucosal lymphocytes are crucial in regulating maintenance intestinal function and immune response [4], [31]. KGF can expand thymic epithelium cells (TECs) and intestinal epithelial cells (ECs) [15], [32] and has been reported to increase IL-7 production in treated mice [15], [32], and also potently augments thymopoiesis and protects from thymic and intestinal damage [15], [32] by signaling via FGFR2IIIb [15], [29], [33]-[35]. Meanwhile, it is believed that IL-7 has effects on developing and mature lymphocytes, and is essential for the ongoing maintenance of the IEL growth and function. In our previous study, we found that IL-7 and KGFR were both expressed in the intestinal epithelial cells (IECs), and KGF could up regulate the IL-7 expression both *in vivo and in vitro* [15]. Through ELISA assay, we also found that KGF significantly increased IL-7 protein expression. When the KGFR was blocked, the above findings were absent [15]. These results suggest that KGF could up-regulate the IL-7 expression through interacting with KGFR pathway in IECs. However, the further mechanism which is involved in transmitting extracellular signals to the nucleus remains unknown.

KGF is a multifunctional cytokine, and it would not be surprising if this growth factor initiates different signals to modulate effects on different epithelial cells. A report of signaling pathways used by KGF in corneal epithelial cells show that the p42 and p44 MAPKs are activated by KGF in human corneal epithelial cells [36]. In this study, our studies were directed toward identifying the signaling molecules activated by KGF to mediate effects on intestinal epithelial cell functions. We found that KGF activated STAT1 in human intestinal epithelial cells, which was the first report of the STAT1 signaling pathways involved by KGF in intestinal epithelial cells. We found KGF increased P-Tyr-STAT1 but not STAT1 in LoVo cells, and P-Tyr-STAT1expression was decreased by blocking agents used, including RPM and AG490. RPM is a *streptomyces* derivative that is critical for the regulation of cell growth, cell proliferation, cell motility and cell survival [37]. More importantly, other data directly support the idea that RPM inhibits the activity of STAT1 [38]. Furthermore, AG490 is an inhibitor of the JAK-2, JAK-3/STAT signaling pathway and potently inhibits cytokine-independent cell growth *in vitro* [39]. In the present study, treatment with RPM and AG490 inhibited the activity of STAT1 and the IL-7 mRNA and protein expression in KGF-stimulated LoVo cells, which suggested KGF regulated IL-7 though the STAT1 signaling pathway. The binding of KGF to its receptor results in the activation of receptor-associated phosphorylation of STAT1, and phosphorylated STAT1 forms homodimers, which migrate to cell nucleus and activate transcription.

Interferon regulatory factor-1 and -2 (IRF-1 and -2) are two structurally related members of the IRF family of transcription factors, which are both involved in signal transducing. IFN-γ regulated CIITA pIV by activating transcription (STAT1), which binds to IFN regulatory factor IRF-1 and IRF-2 to an IFN regulatory factor-element (IRF-E) [22]. The role of IRFs in the regulation of IL-7 expression has been explored previously [1], and this work sheds new light on the role of IRF-1 and IRF-2 in the transcriptional regulation of IL-7 by KGF in intestine *in vivo and in vitro*. We found a significantly increased IRF-1 and IRF-2 expression in the total proteins and in the nucleus, which were detected by Western blot and immunofluorence assay, respectively. We also found KGF significantly increased the number of positive cells which express IRF-1 and IRF-2 in the nucleus by immunohistochemistry staining in the mice intestine. In addition, decreased IL-7 mRNA and protein expressions were observed in LoVo cells by obvious suppression of IRF-1 and IRF-2 expression respectively, even following KGF treatment. The studies reported suggest that STAT1 and IRF transcription factors, including IRF-1 and IRF-2 contribute to the transcriptional regulation of IL-7 by KGF.

In this study, we found KGF up-regulated IL-7 expression through the STAT1/IRF-1, IRF-2 signaling pathway, which was the first report of regulation of IL-7 by KGF in intestinal epithelial cells. All of these data may suggest the indirect data to support that KGF may play an important role in mucosal immune responses by regulating IL-7 to help to regulate IEL. This is important because these data would shed new light on the potential role of KGF in therapies aiming to enhance the ability of the immune system in intestine.
